This article has been retracted.

# Role of ESAT-6 in renal injury by regulating microRNA-155 expression via TLR4/MyD88 signaling pathway in mice with *Mycobacterium tuberculosis* infection

**DOI:** 10.1042/BSR20170021

**Published:** 2017-07-27

**Authors:** Zhong-Qi Zhou, Zhi-Kui Wang, Lei Zhang, Yue-Qin Ren, Zhong-Wei Ma, Nan Zhao, Fu-Yun Sun

**Affiliations:** 1 Department of Nephrology, Linyi People’s Hospital, Linyi 276003, P.R. China; 2 Department of Second Nephrology, Cangzhou Central Hospital, Cangzhou 061000, P.R. China

**Keywords:** Early secretory antigenic target-6, MicroRNA-155, Myeloid differentiation factor 88, Mycobacterium tuberculosis, Renal injury, Toll-like receptor 4

## Abstract

The study aims to investigate the underlying mechanism involved in the early secretory antigenic target-6 (ESAT-6) in renal injury through regulation of the expression of *miR-155* through the oll-like receptor (TLR)-4 (TLR4)/myeloid differentiation factor 88 (MyD88) signaling pathway in *Mycobacterium tuberculosis* (MTB)-infected mice. Sixty C57BL/6 mice with MTB-induced renal injury were randomly assigned into control, MTB, mimic, inhibitor, inhibitor + ESAT6, and inhibitor + ESAT6 + TAK242 groups. Body weight, the ratio of kidney weight to body weight (Kw/Bw), blood urea nitrogen (BUN), and serum creatinine (Scr) of mice were measured. Flow cytometry was used to detect renal activation in mice. Expressions of *miR-155* and ESAT6 were detected by quantitative real-time PCR (qRT-PCR), and Western blotting was used to examine the expressions of ESAT6, TLR4, and MyD88. Expressions of tumor necrosis factor-α (TNF-α), interleukin-17 (IL-17), and interferon-γ (IFN-γ) were measured by qRT-PCR and ELISA. Compared with the control group, the BUN and Scr levels as well as the expression levels of *miR-155*, TLR4, MyD88, TNF-α, IL-17, and IFN-γ increased, while Kw/Bw decreased in the MTB and mimic groups. In comparison with the MTB group, the above indexes except Kw/Bw were elevated in the mimic group, but were reduced in the inhibitor group, while the Kw/Bw dropped in the mimic group but increased in the inhibitor group. Compared with the inhibitor group, the Kw/Bw decreased while the rest of the indexes increased in the inhibitor + ESAT6 group. ESAT6 may induce renal injury by promoting *miR-155* expression through the TLR-4/MyD88 signaling pathway in MTB-infected mice.

## Introduction

Renal injury, also known as kidney injury, is featured by the progressive degradation in relation to renal function. In addition, the decline of glomerular filtration rate (GFR) that accompanies renal injury consequently results in the deposition of urea and various other chemicals into the blood [1]. Approximately 245000 cases of renal injury occur worldwide each year. Renal injuries have been reported to be the most frequently occurring genitourinary injury [2,3]. Renal injury is pathologically characterized by increased levels of acid, potassium and phosphate, elevated fluid in the body, descending level of calcium, and anemia in later stages [4]. The risk factors of renal injury include age, blood glucose, and patients with reduced baseline renal function tend to develop renal injury [5]. Besides, renal injury can be also caused by blunt trauma, such as motor vehicle collisions and falls [3]. The most common treatment for renal injury is renal replacement therapy and cell-based therapy, correction of uremia-associated factors and protein restriction are also therapeutic options [6,7]. Recently, early secretory antigenic target-6 (ESAT-6) was found to be a promising treatment of renal injury [4].

ESAT-6, secreted by *Mycobacterium tuberculosis* (MTB), has been suggested to be a promising vaccine candidate and it has interference in innate immune response to invading mycobacteria [8]. Due to its ability to combine with laminin and cause lysis of lung epithelial cells, ESAT-6 has been indicated to contribute to the dissemination of MTB [9]. Former studies found that ESAT-6 is associated with elevation of *miR-155* expression [10,11]. *MiR-155* was detected in immune cells and earlier studies have investigated its role in immune cells through the physiological functions [12]. *MiR-155* is associated with up-regulation of inflammatory response and pro-inflammatory increases in *miR-155* expression [13]. A recent study found that the deficiency of *miR-155* is associated with alleviation of renal injury [14]. As one of the best pathogen detector, toll-like receptors (TLRs) play an important role in both innate and adaptive host immune responses by binding to ligands in pathogens [15]. TLR4, a member of TLR family, exists in cell membrane and cytoplasm and is studied in immune cells [16]. Myeloid differentiation factor 88 (MyD88) is a kind of adaptor protein which plays a role in signal transduction through most TLRs and IL-1 receptor (IL-1R)/IL-18 receptor (IL-18R) family [17]. A former study showed that mice deficient in TLR4 and MyD88 are less affected by bacteria, providing evidence that the inhibition of TLR-4/MyD88 signaling pathway attenuates renal injury [18]. In the present study, we aimed to explore how ESAT-6 affected renal injury through investigating its interaction with *miR-155* via TLR-4/MyD88 signaling pathway, which is expected to pave the way for the regimen of renal injury.

## Materials and methods

### Ethics statement

All animal procedures were conducted with approval from the Experimental Animal Ethics Committee of Linyi People’s Hospital. All experiments were carried out in strict accordance with the guidelines on the protection and use of animals in International Association for the Study of Pain [19].

### Experimental animals

This experiment was conducted on 60 C57BL/6 mice (30 males and 30 females), weighing 18–22 g and ageing 6–8 weeks, purchased from Shanghai SLAC Laboratory Animal Co., Ltd (Shanghai, China). The mice were kept in a clean grade animal house at 22°C, with free access to water and food.

### Preparation for MTB strain and establishment of renal injury model

MTB H37R strain (number: 9302025), purchased from Beijing Strain Preservation Center of China Institute of Drug Control, was incubated in 7H11 slant solid medium at 37°C for 21 days and then transferred to 7H9 liquid medium for 4-week culture. After that, bacterial fluid was collected, centrifuged at 3800 rpm for 15 min and diluted into suspension in RPMI-1640 medium with 10% FBS but without antibiotic, and its concentration was adjusted to 5 × 10^6^ CFU. Each mouse was caused renal injury by injecting with 5 × 10^6^ CFU of MTB H37Ra in tail vein. The mice were divided into six groups, with ten mice in each group: control group, MTB group, mimic group, inhibitor group, inhibitor + ESAT6 group, and inhibitor + ESAT6 + TAK242 group. The treatment regimens are presented in Table 1. Recombinant protein ESAT6 was purchased from Nanjing Sai Hongrui Biotech Company (number: PRO-563) as immunizing antigen (dose: 50 μg/kg). *MiR-155* mimic (number: PM12601) and *miR-155* inhibitor (number: AM12601) were both bought from Ambion company. Each mouse was infected by tail-vein injection with 0.5 ml mimics, inhibitor, and ESAT6 using EntransterTM-*in vivo* kit (number: 18668-11-1) only once during the experiment.

**Table 1:** Treatment regimens for mice amongst groups

Group	*n*	Treatment scheme
Control	10	Untreated
MTB	10	Tail-vein injection with MTB
Mimic	10	Tail-vein injection with MTB and *miR-155* mimic
Inhibitor	10	Tail-vein injection with MTB and *miR-155* inhibitor
Inhibitor + ESAT6	10	Tail-vein injection with MTB, *miR-155* inhibitor, and recombinant protein ESAT6
Inhibitor + ESAT6 + TAK242	10	Tail-vein injection with MTB, *miR-155* inhibitor, recombinant protein ESAT6, and TAK242

### Sample collection

In the eighth week of experiment, the mice in each group were put in clean metabolic cages and their urine and blood samples were obtained and then preserved at −80°C for spare. Mice were weighed and anesthetized with 3% pentobarbital sodium (Sigma–Aldrich Chemical Company, St. Louis, Missouri, U.S.A.). After being killed, their right kidneys were weighed and the ratio of kidney weight to body weight (Kw/Bw) was calculated. Some renal tissues were preserved in refrigerator with a temperature of −80°C. Other renal tissues were fixed by 4% folmalin, dehydrated in gradient ethanol, embedded in paraffin, and cut into 5-μm thick tissue sections.

### Measurement of renal function

Levels of blood urea nitrogen (BUN) and Cr were detected using the urease continuous monitoring method and picric acid method, respectively. The reagent was made according to the instructions of kits purchased from Shanghai Rongsheng Biotech Company (Shanghai, China). The detection of serum creatinine (Scr) level adopted picric acid method, which was made following instructions on the use of reagent kits from Shanghai Rongsheng Biotech Company. Absorbance (A1) at 30 s and absorbance (A2) at 90 s in each tube were recorded. The respective levels were calculated using the following formula: BUN (mmol/l) = (sample to be tested (A2) – sample to be tested (A1))/(calibration solution (A2) – calibration solution (A1)) × calibration solution concentration.

### ELISA

The ELISA kit was purchased from eBioscience, San Diego, California, U.S.A. The sample (100 μl) to be tested was incubated at 37°C for 90 min. After washing, biotinylated antibody working fluid (100 μl) was added, and further incubation was performed at 37°C for 60 min. Next, 100 μl of present enzyme-bound reactants (light away) working liquid was added and incubated at 37°C for 30 min after washing. Following these, plates was washed three times, and 100 μl of substrate was added and incubated at 37°C for 15 min (light away). The optical density (OD) value of each tube was measured at 450 nm using microplate reader (BioTek Synergy 2). Standard curve was drawn according to OD values and was analyzed to calculate the levels of tumor necrosis factor-α (TNF-α), interleukin-17 (IL-17), and interferon-γ (IFN-γ) in plasma of mice amongst the groups.

### Hematoxylin and Eosin staining

Paraffin sections of renal tissues were dewaxed with xylene, hydrated with gradient alcohol, dyed with Hematoxylin for 10 min, and rinsed with water. Then they were differentiated in hydrochloric acid alcohol for 30 s, blued by ammonia for 30 s, rinsed with water twice, counterstained with Eosin solution for 3 min, dehydrated with alcohol, transparentized with xylene, and sealed with neutral resin. The histopathological changes in tissue sections were observed using an optical microscope (CX31, Olympus, Japan). Four fields of view were randomly selected in each section and photographed, and the average value was calculated. All kits were purchased from Boster Bioengineering Co. Ltd., Wuhan, China.

### Sirius Red staining

Sirius Red staining was used to observe interstitial collagen fibers. Paraffin sections of renal tissues were dewaxed with xylene, hydrated with gradient alcohol (Boster Bioengineering Co. Ltd., Wuhan, China), washed with distilled water for three times, dyed with saturated Picric acid-Sirius Red (10 ml of 0.5% Sirius Red, 90 ml picric saturated liquid) for 30 min, differentiated and dehydrated with absolute ethanol, transparentized with xylene, and sealed with neutral resin. The deposition of collagen fibers in renal tissues was observed. Semiquantitative analysis was conducted on deposition of collagen fibers in renal tissues of C57BL/6 mice by the utilization of Sirius Red staining sections [20]. The linear deposition of collagen fibers on glomerulus vessel wall, glomerulus cyst wall, and basement membrane of renal tubular epithelial cells was recorded as 0. The funicular and taeniform deposition of collagen fibers around glomerulus and small vessels was recorded as 1. A moderate amount of taeniform and funicular deposition of collagen fibers around glomerulus and small vessels or a small amount of funicular deposition of collagen fibers in renal interstitium was marked as 2. Finally, 3 referred to a large amount of funicular and taeniform deposition of collagen fibers around glomerulus and small vessels, or funicular and taeniform deposition of collagen fibers in renal interstitium. The deposition of interstitial collagen fibers was analyzed based on semiquantitative analysis results. The quantitative analysis was done using a blind method, namely, group names and information was not available to investigators.

### Quantitative real-time PCR

Total RNA was manually extracted from renal tissues of mice by using TRIzol (15596026, Invitrogen, U.S.A.) following the instructions of miRNeasy Mini Kit (217004, Qiagen, Hilden, Germany). The concentration and purity of RNA samples were determined using the NanoDrop2000 (NanoDrop2000c, Thermo, U.S.A.), and the samples were preserved at −80°C. According to the gene sequence published in GenBank database, the PCR primers were designed using Primer 5.0 primer design software by Shanghai Jima Co., Ltd. (Shanghai, China) (Table 2). The quantitative real-time PCR (qRT-PCR) reaction was performed using ABI PRISM 7500 real-time PCR system (ABI, U.S.A.) and SYBR Green I Fluorescent Assay kit (DRR041A, Takara). U6/glyceraldehyde 3-phosphate dehydrogenase (GAPDH) was taken as an internal control, relative expression of targetted gene was calculated by 2^−ΔΔ^*C*_t_ [21]: Δ *C*_T_ = *C*_T_ (target gene) – *C*_T_ (reference gene), ΔΔ *C*_t_ = Δ *C*_t_ (experiment group) – Δ *C*_t_ (control group).

**Table 2:** Primer sequences for qRT-PCR

Gene		Sequences (5′-3′)
*miR-155*	RT primer	5′-GTCGTATCCAGTGCAGGGTCCGAGGTATTCGCACTGGATACGACCCCCTA-3′
U6	RT primer	5′-GTCGTATCCAGTGCAGGGTCCGAGGTGCACTGGATACGACAAAATATGGAAC-3′
*miR-155*	Forward	5′-GTGCTGCAAACCAGGAAGG-3′
	Reverse	5′-CTGGTTGAATCATTGAAGATGG-3′
U6	Forward	5′-TGCGGGTGCTCGCTTCGGCAGC-3′
	Reverse	5′-CCAGTGCAGGGTCCGAGGT-3′
ESAT-6	Forward	5′-CGGAATTCGCCACC ATGACAGAGCAGCAGTGG-3′
	Reverse	5′-GCACGCCCCAAGCTTCTATGCGAACATCCCAGT-3′
TNF-α	Forward	5′-CCACCATCAAGGACTCAA-3′
	Reverse	5′-GTCACCAAATCAGCGTTA-3′
IL-17	Forward	5′-GGGAAGTTGGA CCACCACAT-3′
	Reverse	5′- TTCTCCACCCGGAAAGTGAA-3′
IFN-γ	Forward	5′- ACACGCCGCGTCTTGGT-3′
	Reverse	5′- TTCAATGAGTGTGCCTTGGC-3′
TLR4	Forward	5′- TGGATACGTTTCCTTATAAG-3′
	Reverse	5′- GAAATGGAGGCACCCCTTC-3′
MyD88	Forward	5′- CGAGAGCTGGAGCAAACGGAGTTCAAG-3′
	Reverse	5′- GCTGGCTAGTGATGGACCACACGCA-3′
GAPDH	Forward	5′- ACCACAGTCCATGCCATCAC-3′
	Reverse	5′- TCCACCACCCTGTTGCTGTA-3′

RT, reverse transcriptase.

### Western blotting

Tissue protein was extracted and its concentration was detected following the instructions of BCA Kit (Boster Bioengineering Co. Ltd., Wuhan, China). Sample buffer was added to the protein sample and they were boiled at 95°C for 10 min, with 30 μg sample in each well. Proteins were separated by PAGE (10% gel) (Boster Bioengineering Co. Ltd., Wuhan, China). Electrophoresis voltage turned from 80 to 120 V, and the proteins were transferred on to PVDF membrane with a transfer voltage of 100 mV for 45–70 min. After blocking with 5% BSA for 1 h, the membrane was added with diluted primary antibodies (1:1000), including ESAT-6 (ab26246, Abcam, Cambridge, U.K.), TLR4 (ab13556, Abcam, Cambridge, U.K.), MyD88 (ab2068, Abcam, Cambridge, U.K.), β-actin (ab8226, Abcam, Cambridge, U.K.), and kept at 4°C overnight. The PVDF membrane was washed with Tris-buffered saline Tween-20 (TBST) three times (5 min for each time). The corresponding secondary antibody (Abcam, Cambridge, U.K.) was supplemented and incubation was conducted at room temperature for 1 h. PVDF membrane was washed again for three times (5 min each time), and developing was performed with chemiluminescence reagent. GAPDH was used as the internal control, and Bio–Rad Gel Dol EZ imager (Gel Doc EZ Imager, Bio–Rad, California, U.S.A.) was used for developing. The gray level of target protein band was calculated through ImageJ Software.

### Statistical analysis

Data analysis was conducted using SPSS21.0 software (SPSS Inc., Chicago, IL, U.S.A.). Experiment was repeated over three times, and the mean and S.D. were calculated. The measurement data were expressed as mean ± S.D. The *t*test was used for comparison between two groups, and one-way ANOVA was performed for comparison amongst multiple groups. ANOVA was used in the event of homogeneity of variance. Wilcoxon’s rank sum was used in heterogeneity of variance. Pearson analysis was performed for gene correlation. *P*-value of less than 0.05 was denoted with statistical significance.

## Results

### Body weight and Kw/Bw of mice amongst the control, MTB, mimic, inhibitor, and inhibitor + ESAT6 groups

Body weight and Kw/Bw of mice were analyzed (Table 3). The results revealed that before experiment, there was no remarkable difference in body weight of C57BL/6 mice amongst the five groups. After experiment, compared with the control group, the body weight significantly decreased in the MTB, mimic, and inhibitor + ESAT6 groups, while the kidney weight and Kw/Bw increased (all *P*<0.05). There were no obvious differences between the inhibitor group and control group (all *P*>0.05). In comparison with the MTB group, the body weight reduced in the mimic group but increased in the inhibitor group, and the kidney weight and Kw/Bw increased in the mimic group but decreased in the inhibitor group (all *P*<0.05). Compared with the inhibitor group, the body weight decreased while kidney weight and Kw/Bw increased in the inhibitor + ESAT6 group (all *P*<0.05), and there was no significant difference between the inhibitor + ESAT6 + TAK242 and the inhibitor group (*P*>0.05). The results suggested that the body weight decreased while the Kw/Bw increased in MTB-infected mice. By promoting *miR-155* expression, ESAT-6 plays a role in the reduction in Kw/Bw.

**Table 3:** Comparisons of body weight and the Kw/Bw of mice amongst the groups

Group	Weight before experiment (g)	Weight after experiment (g)	Kidney weight after experiment (mg)	Kw/Bw
Control	19.78 ± 1.20	29.59 ± 0.79	0.44 ± 0.06	1.40 ± 0.20
MTB	19.65 ± 0.91	25.88 ± 1.15*	0.50 ± 0.02*	1.94 ± 0.09*
Mimic	19.42 ± 1.17	22.49 ± 1.39*^†^	0.59 ± 0.03*^†^	2.63 ± 0.21*^†^
Inhibitor	19.56 ± 1.10	29.13 ± 1.20^†^	0.43 ± 0.05^†^	1.48 ± 0.21^†^
Inhibitor + ESAT6	19.33 ± 1.24	25.36 ± 1.27*^‡^	0.51 ± 0.03*^‡^	2.02 ± 0.17*^‡^
Inhibitor + ESAT6 + TAK242	19.63 ± 1.15	29.07 ± 1.13^†^	0.41 ± 0.04^†^	1.45 ± 0.18^†^

*, compared with the control group, *P*<0.05; ^†^, compared with the MTB group, *P*<0.05; ^‡^, compared with the inhibitor group, *P*<0.05.

### Pathological changes and renal function of renal tissues in mice amongst groups

Figure 1A showed the pathological changes in renal injury in mice of each group. In the control group, glomerular and renal tubules were in normal structure, and there was no denaturation, necrosis, and inflammatory cell infiltration. The MTB group demonstrated slight increase in the mesangial matrix, vacuole in renal tubular epithelial cells, narrowing of renal tubular, and inflammatory cell infiltration in renal interstitium. In the mimic group, mesangial matrix was slightly increased, renal tubular epithelial cells showed vacuole and swelling, the brush border disappeared, and a large amount of inflammatory cell infiltration was present in renal interstitium. The inhibitor group showed no increase in mesangial matrix but a little inflammatory cell infiltration. The inhibitor + ESAT6 group showed slight increase in mesangial matrix, swelling in renal tubular, vacuole in renal tubular epithelial cells, and inflammatory cell infiltration in renal interstitium. The results suggested that renal injury was caused by MTB infection, protection against renal injury can be achieved through inhibiting the expression of *miR-155*, and ESAT-6 aggravated renal injury by increasing expression of *miR-155*. Changes in Scr and BUN indicated that the levels of BUN and Scr increased in the MTB, mimic and inhibitor + ESAT-6 groups when compared with the control group (all *P*<0.05). In comparison with the MTB group, the levels of BUN and Scr elevated in the mimic group but reduced in the inhibitor group (all *P*<0.05). Compared with the inhibitor group, the levels of BUN and Scr were up-regulated in the inhibitor + ESAT-6 group (all *P*<0.05). There was no significant difference in the levels of BUN and Scr between the inhibitor + ESAT-6 + TAK242 and the inhibitor groups (Figure 1B,C). The results suggested that the levels of BUN and Scr were increased in MTB-infected mice and the down-regulation of *miR-155* could reduce the levels of BUN and Scr through the TLR4 signaling pathway.

**Figure 1:** Comparisons of pathological changes of renal tissues of mice amongst groups (**A**) HE (Hematoxylin and Eosin) staining of renal tissues amongst groups (×400); (**B**) detection of BUN; (**C**) detection of Scr; *, compared with the control group, *P*<0.05; #, compared with the MTB group, *P*<0.05; &, compared with the inhibitor group, *P*<0.05.

### Deposition of renal interstitial collagen fibers amongst groups

In the control group, there was a small amount of deposition of collagen fibers on renal capsule wall, basement membrane of glomerulus, and basement membrane and vessel of renal tubular epithelial cells. The MTB group showed a moderate amount of taeniform and funicular deposition of collagen fibers around glomerulus and small vessels, and a small amount of funicular deposition of collagen fibers in renal interstitium. The mimic group showed a large amount of funicular and taeniform deposition of collagen fibers around glomerulus and small vessels, and in renal interstitium. There was a small amount of funicular deposition of collagen fibers around glomerulus and small vessels in the inhibitor group. In the inhibitor + ESAT6 group, there was a large amount of funicular deposition of collagen fibers on renal capsule wall and around glomerulus and small vessels. The results (Figure 2) revealed that the deposition of collagen fibers could be caused by MTB infection. Reducing the deposition of collagen fibers can be achieved through decreasing expression of *miR-155* via the TLR4 signaling pathway.

**Figure 2:** Comparisons of deposition of renal interstitial collagen fibers of mice amongst groups (×400) *, compared with the control group, *P*<0.05; #, compared with the MTB group, *P*<0.05; &, compared with the inhibitor group, *P*<0.05.

### Expression of *miR-155* and ESAT6 of renal tissue amongst groups

Results of expressions of *miR-155* and ESAT6 were detected by qRT-PCR and Western blotting showed that compared with the control group, the expressions of *miR-155* and ESAT6 increased in the MTB, mimic, and inhibitor + ESAT6 groups (all *P*<0.05). In comparison with the MTB group, the expressions of *miR-155* and ESAT6 increased in the mimic group but decreased in the inhibitor group (all *P*<0.05). Compared with the inhibitor group, the expressions of *miR-155* and ESAT6 increased in the inhibitor + ESAT6 (*P*<0.05), while there was no significant difference in the inhibitor + ESAT6 + TAK242 group (Figure 3A–D). Based on the results shown in Figure 3E, expression of *miR-155* was positively connected with expression of ESAT6 (*P*<0.05).

**Figure 3:** Expression of *miR-155* and ESAT6 amongst groups (**A**) Expression of *miR-155* in renal tissue; (**B**) mRNA expression of ESAT6; (**C**) protein band of ESAT6 in renal tissue; (**D**) quantization histogram of protein expression of ESAT6; (**E**) correlation of *miR-155* and ESAT6; *, compared with the control group, *P*<0.05; #, compared with the MTB group, *P*<0.05; &, compared with the inhibitor group, *P*<0.05.

### mRNA and protein expression of TLR4/MyD88 signaling pathway related proteins amongst groups

The mRNA and protein expressions of TLR4/MyD88 were displayed in Figure 4. Compared with the control group, the expressions of TLR4 and MyD88 increased in the MTB, mimic, and inhibitor + ESAT6 groups (all *P*<0.05). In comparison with the MTB group, the expressions of TLR4 and MyD88 increased in the mimic group but decreased in the inhibitor group (all *P*<0.05). Compared with the inhibitor group, the expressions of TLR4 and MyD88 increased in the inhibitor + ESAT6 group (all *P*<0.05), while there was no difference found in the inhibitor + ESAT-6 + TAAK242 group. The results suggested that the expressions of TLR4 and MyD88 were elevated in MTB-infected mice, and ESAT-6 promoted the *miR-155* expression to increase the expressions of TLR4 and MyD88.

**Figure 4:** Protein expression of TLR4 amongst groups (**A**) The mRNA expression of TLR4 in each group detected by qRT-PCR; (**B**) the protein expressions of TLR4 and MyD88 in each group detected by Western blotting; (**C**) the changes of protein expressions of MyD88 and TLR4 in each group detected by gray analysis; *, compared with the control group, *P*<0.05; #, compared with the MTB group, *P*<0.05; &, compared with the inhibitor group, *P*<0.05.

### mRNA and protein expression of inflammatory cytokines amongst groups

Compared with the control group, the mRNA and protein expressions of cytokines TNF-α, IL-17, and IFN-γ increased in the MTB, mimic, and inhibitor + ESAT6 groups (all *P*<0.05). In comparison with the MTB group, the mRNA and protein expressions of TNF-α, IL-17, and IFN-γ increased in the mimic group but decreased in the inhibitor group (all *P*<0.05). Compared with the inhibitor group, the mRNA and protein expressions of TNF-α, IL-17, IFN-γ increased in the inhibitor + ESAT6 group (all *P*<0.05). No significant differences were observed between the inhibitor + ESAT6 + TAK242 group and the inhibitor grop (Figure 5). The results clarified that ESAT-6 enhanced the expressions of TNF-α, IL-17, and IFN-γ by promoting *miR-155* expression through TLR4 signaling pathway in MTB-infected mice.

**Figure 5:** Expressions of inflammatory factors amongst groups (**A**) mRNA expression of TNF-α in each group detected by qRT-PCR; (**B**) mRNA expression of IFN-γ in each group detected by qRT-PCR; (**C**) mRNA expression of IL-17 in each group detected by qRT-PCR; (**D**) expression of TNF-α in each group detected by ELISA; (**E**) expression of IFN-γ in each group detected by ELISA; (**F**) expression of IL-17 in each group detected by ELISA; *, compared with the control group, *P*<0.05; #, compared with the MTB group, *P*<0.05; &, compared with the inhibitor group, *P*<0.05.

## Discussion

In the present study, we investigated the effect of ESAT-6 on renal injury by establishing MTB-infected mouse models. The results showed that groups infected by MTB appeared with renal injury, demonstrating that ESAT-6, secreted by MTB, promoted the development of renal injury by up-regulating the expression of *miR-155* to activate the TLR4/MyD88 signaling pathway.

Our study showed that MTB infection caused the renal injury in mice. Kidney is a good colonization area for MTB and mainly conducts its proliferation in the medullary region, where it can build cortical granulomas and damage local tissues through the build-up of cortical granulomas [22]. Davies et al. found that patients with renal disease are at an increased risk of tuberculosis (TB), especially those with chronic kidney disease (CKD) [23]. MTB, a kind of intracellular pathogen and the main cause of TB, establishes infection through inhibition of phagosome maturation, as well as preventing the consequences from delivering to the lysosome and rendering its surrounding environment more suitable for bacterial survival and replication [24]. Recently, extrapulmonary MTB has been found to cause renal injury [25]. After being infected with MTB, the body weight of mice decreased while Kw/Bw increased. This was in consistence with former studies, where a reduction in body weight was followed by an elevation of Kw/Bw in mice with renal injury [26,27]. MTB-infected mice showed increased levels of BUN and Scr, which indicated that renal injury is characterized by higher levels of BUN and Scr. This was confirmed by previous studies that the levels of BUN and Scr were elevated in mice with renal injury [28–30]. MTB group displayed a slight increase in the mesangial matrix, vacuole in renal tubular epithelial cells, narrowing of renal tubular and inflammatory cell infiltration in renal interstitium. Previous studies have also demonstrated that renal injury was pathologically featured by expansion of the mesangial matrix, increasing patches of tubular vacuolation, brush border loss, and infiltration of inflammatory cells in the renal interstitium [31,32]. MTB-infected mice presented moderate amount of band and strand collagen fibers around glomerulus and small vessels, and small amount of collagen fibers in renal interstitium, which revealed existence of collagen fiber deposition in renal injury [33,34].

In addition, MTB group showed higher *miR-155* expression than the control group, which indicated that higher *miR-155* expression is related to renal injury. Additionally, miRNAs are closely linked to the pathogenesis of diabetic nephropathy [35]. *MiR-155* is a kind of inflammation-associated miR and connected positively with GFR [36]. During innate immune response, autoimmune disorders and a variety of malignancies, expression of *miR-155* increase in renal disease [37]. Former studies demonstrated that *miR-155* expression was up-regulated in renal disease [35,38]. Qi et al. [39] proved that dioscin alleviates lipopolysaccharide-induced inflammatory kidney injury through the miRNA TLR4/MyD88 signaling pathway. Renal ischemia/reperfusion injury was attenuated through inhibition of TLR4/MyD88 signaling pathway [40]. Li et al. [41] also demonstrated that increased *miR-155* expression activates the TLR3/TLR4 signaling pathways, and the decreased *miR-155* expression inhibits these pathways. Thus, we hypothesized that *miR-155* is positively associated with the activation of TLR4/MyD88 signaling pathway in renal injury, which was supported by our results that the increased expressions of TLR4 and MyD88 were found in the MTB and mimic groups in contrast with the control group, and the mimic group was higher than the MTB group.

Furthermore, higher levels of *TNF-α, IL-17*, and *IFN-γ* mRNA and protein expressions were observed in MTB, mimic, and inhibitor + ESAT6 groups in comparison with the control group. Inflammatory factors were used as biomarkers to determine renal injury [42]. Lin et al. [43] found that TLR4 and its adaptor MyD88 may have a positive effect on enhancing the expressions of IL-1β and TNF-α, from which we hypothesized that elevated expression of inflammatory factors are correlated with activation of TLR4/MyD88 signaling pathway. The *miR-155* expression was higher in inhibitor + ESAT6 group in comparison with the inhibitor group, indicating a stimulatory role of ESAT-6 in *miR-155* expression. ESAT6 may contribute to cellular invasion, escape from phagolysosomes, cell-to-cell spread and dissemination of MTB by acting like a cytolytic pore-forming toxin [44]. ESAT-6 secreted by MTB is not only characterized by virulence, but also demonstrates a strong immunotherapeutic potential to fight against MTB [45]. *MiR-155* has the highest expression of miRNA during MTB infection and its up-regulation is directly linked to ESAT-6 [11]. In the present study, it was hypothesized that ESAT-6 promoted *miR-155* expression, which was in consistence with former scientific findings that ESAT-6 plays a role in the elevation of *miR-155* expression [10,11].

## Conclusion

In conclusion, the results of the study and evidence suggest that ESAT-6 may contribute to renal injury of MTB-infected mice by promoting *miR-155* expression through the TLR4/MyD88 signaling pathway. The data implied that ESAT-6 is expected to be a potential target for therapy of renal injury. However, as to whether the inhibitors and mimics appear to act locally in the kidney and whether both of them have an effect on other paracrine pathways is in need of further scientific investigation. As relatively few studies have been conducted on the role of ESAT-6 in renal injury on a molecular basis, further larger scale trials and investigations are needed to further perfect this work.

## Abbreviations

BUN: blood urea nitrogen
ESAT-6: early secretory antigenic target-6
GAPDH: glyceraldehyde 3-phosphate dehydrogenase
GFR: glomerular filtration rate
IL-17: interleukin-17
IFN-γ: interferon-γ
Kw/Bw: ratio of kidney weight to body weight
MTB: *Mycobacterium tuberculosis*
MyD88: myeloid differentiation factor 88
qRT-PCR: quantitative real-time PCR
Scr: serum creatinine
TB: tuberculosis
TLR: toll-like receptor
TNF-α: tumor necrosis factor-α
